The article "A Deep Ranking Weighted Multihashing Recommender System for Item Recommendation" was published in 2022. Journal: Comput Intell Neurosci.

# A Deep Ranking Weighted Multihashing Recommender System for Item Recommendation

**DOI:** 10.1155/2022/7393553

**Published:** 2022-10-10

**Authors:** Suresh Kumar, Jyoti Prakash Singh, Vinay Kumar Jain, Avinab Marahatta

**Affiliations:** ^1^Department of Computer Science and Engineering, NIT Patna, India; ^2^Department of Management (PG), MIT World Peace University, Pune, India; ^3^Center for Multidisciplinary Studies and Innovation (CeMuSI), Kathmandu, Nepal

## Abstract

Collaborative filtering (CF) techniques are used in recommender systems to provide users with specialised recommendations on social websites and in e-commerce. But they suffer from sparsity and cold start problems (CSP) and fail to interpret why they recommend a new item. A novel deep ranking weighted multihash recommender (DRWMR) system is designed to suppress sparsity and CSP. The proposed DRWMR system contains two stages: the neighbours' formation and recommendation phases. Initially, the data is fed to the deep convolutional neural network (CNN). The significant features are extracted from CNN. The CNN contains an additional layer; the hash code is generated by minimising pairwise ranking loss and classification loss. Therefore, a weight is assigned to different hash tables and hash bits for a recommendation. Then, the similarity between users is obtained based on the weighted hammering distance; the similarity between users helps to form the neighbourhood for the active user. Finally, the rating for unknown items can be obtained by taking the weighted average rating of the neighbourhood, and a list of the top *n* items can be produced. The effectiveness and accuracy of the proposed DRWMR system are tested on the MovieLens 100 K dataset and compared with the existing methods. Based on the evaluation results, the proposed DRWMR system gives precision (0.16), the root mean squared error (RMSE) of 0.73 and the recall (0.08), the mean absolute error (MAE) of 0.57, and the *F* − 1 measure (0.101).

## 1. Introduction

Recommendation systems (RS) have recently become common on numerous websites, recommending movies, e-commerce, music, and television programs [1]. Based on the information provided by the user, the RS recommends items for purchase [2]. Several RS have been introduced to predict the behaviour of users and provide better recommendations [3, 4]. In general, RS recommends, based on the individual interests of the user and their previous usage history, finding items with the highest preference [5]. RS is a great machine learning system to increase product sales [6, 7]. Recommendation helps the user to speed up the search process and makes it simple for them to obtain content that is interesting to them, as well as provide them with offers they would not have searched for [8, 9]. Furthermore, companies may attract customers by showing movies and TV shows relevant to their profiles [10].

The approaches to recommendation may be categorised as collaborative filtering (CF), content-based (CB), and hybrid based on the type of data gathered and how it is used in the RS [11]. CB filtering is frequently used in the RS design, which uses items' content to select general characteristics and qualities that suit the user profiles [12]. Then, users compare items to previously liked items and recommend the best matching-items. The CF system works based on a user-item relationship. Hybrid systems utilise both forms of information to prevent issues that arise when only one type is used.

Although the recommendation system has demonstrated its usefulness in various fields, it faces some problems: sparsity and cold start problems (CSP). As the name implies, a sparsity problem develops when customers do not rate an item while purchasing online, resulting in a sparsity of available ratings. The CF method goes through this problem because it uses a rating matrix. A CSP arises when a new product is added to the recommendation system, and no past ratings for that product are available. As a result, an RS must provide options for new users, which makes the accuracy of the recommendations low. Several research groups are working to develop an efficient and well-organised RS algorithm. The methods like local sensitive hashing (LSH) [13], Bayesian personalized ranking (BPR) [14], Cofi Rank-maximum margin matrix factorization (CRMF) [15], etc. are used for removing sparsity and CSP. However, the existing methods fail to generate deep hashing by minimising classification loss, ranking pairwise, and high storage costs, motivating us to develop an efficient method for recommending items.

### 1.1. Contribution

The following are the research work's contributions:

- The hash code is generated by reducing the classification and pairwise ranking loss, which can handle the users with cold start and sparsity problems.
- A weight is introduced to hash tables and hash bits according to their performance.
- The weighted Hamming distance is used to determine user similarity.
- Bit diversity and similarity preservation are utilised to calculate the hash bit's weight, and the MAP score is used to evaluate the weight-based table-wise.
- The proposed DRWMR system performs better for the item recommendation.

The following is a summary of the paper's structure: Section 2 provides an overview of existing works. Our proposed DRWMR System is explained in Section 3. In Section 4, the proposed method is subjected to experimental analysis. Finally, the paper concludes in Section 5.

## 2. Literature Review

Da'u et al. [16] proposed a deep learning method that uses Aspect-based opinion mining (ABOM) in a recommendation system. This method contains two portions. They are rating predictions and ABOM. In the first portion, we utilised multichannel deep convolutional neural networks for extracting aspects. In the second portion, we add aspect-based ratings into a machine's tensor factorisation to predict overall ratings. This method increases the accuracy of the recommendation system, but the time consumption is more significant.

Ye and Liu [17] introduced Collaborative Topic Regression (CTR) and three novel granulation methods for the recommendation strategy. The three granulation methods are LDA-based, PMF-based, and CTR-based, based on building granular structures and conducting granulation. LDA-based and PMF-based methods are developed to extract granular features from content and feedback information. The CTR-based method is designed to be joined with LDA- and PFM-based methods to produce multilevel recommendation information and interpretable granular features. These methods were introduced to overcome the problem of time cost and decision cost. However, this method does not consider users' dynamic preferences.

Chen et al. [18] offered a Dynamic Decay CF (DDCF) recommendation method based on the user's interest. This method has four stages: clustering of items, identification of the interesting level, specification of the decay function, and preference prediction. In item clustering, similar items are grouped without any predefined parameters. Then, in the second stage, based on the number of ratings and time records in the cluster, we can identify the interesting level of users. In the third stage, decay functions describe the preference evolution at every level. Finally, the similarities between the users are calculated based on the decay rates, and future preferences are predicted. This method accurately predicts the user's interests, but the time consumption is high.

Beg et al. [19] introduced a chaotic based reversible data transform method (CRDTM) for preserving privacy in data mining for the recommendation system. This method will dynamically produce the values of RDT parameters during processing time, but it does not need the parameters during recovery. This method can substitute for the standard RDT algorithm, in which memory and bandwidth are considered significant factors. The RDT algorithm is used in the mobile app recommendation area. This method decreases the execution time, but accuracy is low.

Abbasi-Moud et al. [20] offered a context-aware recommendation system for tourism. It consists of three steps. 'Users' preferences are extracted from their reviews and comments in the first step. In the second step, tourist 'attractions' characteristics are extracted from the tourist reviews. In the third step, recommendations are given based on the 'user's preference and its similarity with the tourist attractions' characteristics and contextual information. The contextual information utilised in this method includes location, weather, user preferences, and time. This method gives high accuracy in tourism recommendation. However, the weather may change according to the season, so it's challenging to make a recommendation.

Zhang et al. [21] introduced a novel hybrid probabilistic matrix factorization method for distinguishing between items' attractiveness and users' preferences for a recommendation. It consists of two sub-divisions. One division attempts to predict the rating scores of users by extracting the user's personal preferences from auxiliary data. Another division attempts to model the textual interest of items for different users. These two sub-divisions are formed into a unified framework using a global objective function. This method gives high accuracy.

Choe et al. [22] offered a hierarchical model based on a recurrent neural network (HMRNN) for considering users' item usage histories in time series and sequences in a recommendation. This method contains two layers: a long-term (LT) and a short-term (ST). The ST sequences are handled by the ST layer, typically found in older ones. The LT layer recollects the data from the preceding ST sequences and distributes it to the lasting time. This method increases the amount of stored user history. However, it does not take the consideration of temporal properties.

## 3. DRWMR System

We propose a novel deep ranking weighted multihashing recommender (DRWMR) system to suppress sparsity and CSP by considering CSP and sparsity issues. This method has two stages: the neighbours' formation and recommendation phases. Initially, the user-item rating data of the user is fed into the neighbours' formation stage, and deep convolutional neural networks are used to extract text features. The deep neural network consists of an additional layer (hash table). The hash codes are produced by reducing the classification loss and pairwise ranking loss. The similarity preservation is preserved by pairwise ranking loss, and the prediction error is minimised by classification loss. Because each hash bit performs differently in the RS, it is not easy to treat them all equally. Therefore, a weight is assigned to different hash tables and hash bits for a recommendation. Then, the similarity between users is obtained based on the weighted Hamming distance—the similarity between users helps to get the neighbourhood formation for the active user. Finally, the rating for unknown items can be obtained by taking the weighted average rating of the neighbourhood and producing a list of the top *n* items.  Figure 1 illustrates the architecture of the proposed DRWMR system.

### 3.1. Neighborhood Formation Phase

The user-item rating data is given to the deep CNN, which is used to extract the features. Then, a hash code is generated by minimising classification loss and ranking pairwise loss. Therefore, a weight is assigned to different hash tables and hash bits. According to weighted Hamming distance, the most similar users are identified as active users.

#### 3.1.1. Deep CNN

The convolution and max pooling layers are used to extract the features. The demographic data of the user is fed to the convolution pooling layer. The convolution pooling layer is formed with the rectified linear activation function in the first three layers. The max pooling process is utilised in the initial convolution pooling layers, and the average pooling process is used in the final convolution pooling layers. They mostly use the original raw data to extract high-level representations. In the first three convolutional layers, we use 32, 32, and 64 with stride 1 for every convolution layer and a kernel size of 5 × 5. 3 × 3is the size for pooling operations, while 2 is the stride for each pooling layer. The fully-connected layer uses a rectified linear activation function and a dropout layer with a 0.5 dropout ratio. A tangent-like activation is used in the hash code layer to output hash codes. The softmax function is utilised as the activation function in the classification layers to preserve semantic similarity. The classification and hash code layers are sequentially learned in every training epoch. In the first fully-connected layer, the unit number is 500, the hash code's length is equal to the second fully-connected layer's output, and the number of classes is similar to the third fully-connected layer's output. A deep CNN architecture is constructed with this framework to learn the function of nonlinear transformation *α*(*∗*) using the input as data. The hash bit is determined by using

(1) $$\begin{array}{c} a=sign\left(\alpha \right.\left(K\right)\text{,} \end{array}$$

where *K* denotes the raw data, and sign (*y*) signifies the sign function.

The deep neural network consists of an additional layer (hash table). The hash codes are produced by reducing the classification loss and pairwise ranking loss. The similarity preservation is preserved by pairwise ranking loss, and the prediction error is minimised by classification loss. For a pair of users, the pairwise-loss function can be defined as follows:

(2) $$\begin{array}{c} S\left(a_{i},a_{j},I_{i,j}\right)=\frac{1}{2}\left(1-I_{i,j}\right)H_{d}\left(a_{i},a_{j}\right)+\frac{1}{2}I_{i,j}\max\;\left(l-H_{d}\left(a_{i},a_{j}\right),0\right)\text{.} \end{array}$$

Such that *a*_*i*_, *a*_*j*_ ∈ {+1, −1}^*h*^,

where *a* denotes the user *K*'s binary hash code, *H*_*d*_(*a*_*i*_, *a*_*j*_) signifies the Hamming distance between *a*_*i*_, an d *a*_*j*_. The similarity between *a*_*i*_ an d *a*_*j*_is denoted by *I*_*i*,*j*_, it is defined as

(3) $$\begin{array}{c} I_{i,j}=\left\{\begin{array}{c} 0\;if\;a_{i},an\;d\;a_{j}\;aresimilar\;\\ 1\;if\;a_{i},an\;d\;a_{j}\;are\;dissimilar \end{array}\right.\text{.} \end{array}$$

The Hamming distance between the input user *e*_*i*_, and its pairwise user is calculated to produce an arranged hamming list. The pairwise ranking loss for an input user *e*_*i*_ is defined in the following equation:.

(4) $$\begin{array}{c} P\left(a_{i}\right)=\overset{M_{i}}{\underset{j=1}{\sum }}P\left(S\right.\left(a_{i},a_{j},I_{i,j}\right)=\overset{M_{i}}{\underset{j=1}{\sum }}S^{2}\left(a_{i},a_{j},I_{i,j}\right)\text{,} \end{array}$$

where *M*_*i*_ denotes the pairwise user's number for user *e*_*i*_. Users similar to *e*_*i*_ should have short Hamming distances, therefore they seem at the top of the arranged Hamming list, whereas dissimilar data seem at the bottom. On the other hand, data at the improper positions of the Hamming list of*e*_*i*_ has substantial loss values. We aim to decrease the overall loss function for a training database with *M* user, which is given in the following equation:

(5) $$\begin{array}{c} P=\overset{M}{\underset{i=1}{\sum }}\overset{M_{i}}{\underset{j=1}{\sum }}P\left(a_{i},a_{j}\right)\text{.} \end{array}$$

Such that *a*_*i*_, *a*_*j*_ ∈ {+1, −1}^*h*^, *i*=1,………*M*.

Since the hash codes are in binary, the fitness function is nondifferentiable. As a result, using the gradient descent approach is challenging for optimising the fitness function. Therefore, to overcome this problem, a tanh approximation function is used instead of the sign function. The tanh-like function can be used to estimate*a*_*i*_'s hash code, which is given as follows:

(6) $$\begin{array}{c} p_{i}\left(a_{i}\right)=\frac{e^{a_{i}}-e^{{-a}_{i}}}{e^{a_{i}}+e^{{-a}_{i}}}\text{.} \end{array}$$

The Euclidean distance *E*_*d*_(*p*_*i*_,)*PJ*between two users, can be further estimated as the Hamming distance *H*(*a*_*i*_, *a*_*j*_) using the calculated hash codes determined in the following equation:

(7) $$\begin{array}{c} E_{d}\left(p_{i},p_{j}\right)={\left\|a_{i}-a_{j}\right\|}_{2}^{2}\text{.} \end{array}$$

A regularisation term is included to reduce the quantisation loss. The final loss function is determined in the following equation:

(8) $$\begin{array}{c} P=\overset{M}{\underset{i=1}{\sum }}\overset{M_{i}}{\underset{j=1}{\sum }}\frac{1}{2}\left\{{\left(I_{i,j}E_{d}\left(p_{i},p_{j}\right)+\frac{1}{2}I_{i,j}\max\;\left(l-E_{d}\left(p_{i},p_{j}\right),0\right)\right)}^{2}\right\}+\overset{m}{\underset{i=1}{\sum }}\alpha {\left\|p_{i}-a_{i}\right\|}_{2}^{2}\text{.} \end{array}$$

Such that *a*_*i*_, *a*_*j*_ ∈ {+1, −1}^*h*^, *i*=1,………*M*,

where *α* denotes the regularisation term's parameter coefficient. The classification layer outputs the recommendation for the category. As a recommendation function, the softmax function is used. The classification loss is determined in the following equation:

(9) Ci=−∑j=1oD^ijeoXij∑k=1oeoXik.

Where *o* and *o*_*x*_ij_ signify the class's number and the recommended output of *j*'s class for user *e*_*i*_.

#### 3.1.2. Weighted Multihashing

A weighted multihash code is used based on the loss in the hamming distance. It multiplies the bitwise weight and table-wise weight to minimise loss. Each hash bit performs differently in the recommendation task, so it is not fair to treat them all the same. Therefore, a weight is assigned to different hash tables and hash bits. Bit diversity and similarity preservation are integrated for the bitwise weighting. The MAP value is utilised for each hash table to compute the weight-based table-wise. The weight-based table-wise and bitwise may change for dissimilar users. This method adjusts the two weights, and their product determines the final weight. The bit *b* in table *r* final weight is defined as follows:.

(10) $$\begin{array}{c} {WT}_{b,r}={WT}_{{bit}_{b}}\times {WT}_{{bit}_{r}.} \end{array}$$

Similarity preservation (*P*) measures a hash bit's semantic similarity. The hash bit *a*_*r*_′*s*similarity preservation (*P*) is calculated in the following equation:

(11) $$\begin{array}{c} Q\left(a_{b}\right)=\frac{1}{2}\left(a_{b}^{\prime }Ia_{b}-U\right)\text{,} \end{array}$$

where *U* signifies the training sample's number, and *a*_*b*_′ signifies the *a*_*b*_'s transpose.

The bit diversity is utilised to calculate the hash bit's performance. The difference between each user's hash bit is crucial for maintaining recommendation efficiency. Therefore, every hash bit must be independent. The correlation between two hash bits is used to determine bit diversity, which can be determined by the above formula.

Initially, a bitwise correlation metric *R*={*r*_*Q*_ij__|*i*, *j*,………*h*} ∈ *Z*^*h*×*h*^ can be generated by calculating *r*_*Q*_ij__ for bit *a*_*i*_ and *a*_*j*_ pair. The bitwise correlation is measured using the Kappa value, which is determined in the following equation:

(12) $$\begin{array}{c} r_{q}=\frac{\emptyset_{1}-\emptyset_{2}}{1-\emptyset_{2}}\in \left[-1,1\right]\text{,} \end{array}$$

where ∅_1_, and ∅_2_ denote the hash bit's probabilities. Eqn can determine the _1_, and ∅_2_ probabilities.

(13) $$\begin{array}{c} \emptyset_{1}=\frac{w+z}{V}\\ \emptyset_{2}=\frac{\left(w+x\right)\left(w+y\right)+\left(y+z\right)\left(x+z\right),}{v^{2}} \end{array}$$

where *w*, *x*, *y*, and *z* denote the nonnegative variables indicating the sample's number that fulfills the relevant row and column requirements. The bit-correlated matrix *M*={*m*_1_,……, *m*_*h*_} ∈ *Z*^1×*h*^ is formed by assigning the correlated coefficient for each bit. Finally, the bit*a*_*r*_'s bit diversity weight is calculated by the following equation:

(14) $$\begin{array}{c} K\left(a_{b}\right)=\frac{1-f_{b}}{2}\text{,} \end{array}$$

where *f*_*b*_ signifies the *b*^th^ bit's correlated coefficient. To generate a final bitwise weight *WT*_bit_*b*__, the terms mentioned above are first adjusted and multiplied, which is determined in the following equation:

(15) $$\begin{array}{c} {WT}_{{bit}_{b}}=Q\left(a_{b}\right)\times K\left(a_{b}\right)\text{.} \end{array}$$

To combine multiple hash tables, table-wise weight (*WT*_bit_*r*__)for each hash table is determined using the mean average precision. It is specified in the following equation:

(16) $$\begin{array}{c} A=\frac{1}{P}\overset{n}{\underset{b=1}{\sum }}\frac{b}{P_{b}}\times {rel}_{b,} \end{array}$$

where *n* signifies the size of the dataset, *P* denotes the similar user's number in the dataset that relates to the checking user, *P*_*b*_ denotes the similar user's number at the top of the dataset.

### 3.2. Recommendation Phase

The neighbours obtained from the previous phase are used to generate a recommendation. This similarity between the active user and its neighbours is utilised to forecast the final rating for an unknown rating of item *i*. In this regard, the ultimate anticipated rating provided by user *u* for any item *i* is calculated as the following:

(17) $$\begin{array}{c} {Pre\;d}_{u,i}^{U}=\begin{array}{cc} {\bar{r}}_{u}+ & \frac{\sum_{u^{\prime }\in N\left(u\right)}sim\left(u,u^{\prime }\right)\times \left(r_{u^{\prime },i}-{\bar{r}}_{u^{\prime }}\right)}{\sum_{u^{\prime }\in N\left(u\right)}sim\left(u,u^{\prime }\right)}\text{,} \end{array} \end{array}$$

where *N*(*u*) is the user's neighbour, *u* and sim(*u*, *u*′) denote the similarity between two users.

The prediction value of each item can be sorted in descending order, and the top n items from this sorted list of items can be recommended to the user.

The similarity between the users can be obtained by the following equation:

(18) $$\begin{array}{c} sim\left(u,u^{\prime }\right)=\frac{\underset{i\in I}{\sum }\left(r_{u,i}-{\bar{r}}_{u}\right)\left(r_{u^{\prime },i}-{\bar{r}}_{u^{\prime }}\right)}{\sqrt{\underset{i\in I}{\sum }{\left(r_{u,i}-{\bar{r}}_{u}\right)}^{2}}\sqrt{\underset{i\in I}{\sum }{\left(r_{u^{\prime },i}-{\bar{r}}_{u^{\prime }}\right)}^{2}}} \end{array}$$

where *I* is the set of items,*r*_*u*,*i*_ rating of given to item *i*by user $u,{\bar{\;r}}_{u}$ average rating of user *u*.

## 4. Experimental Results and Analysis

This section contains the experimental setup and a description of the datasets for comparative analysis.

### 4.1. Dataset Description

The movie Lens 100 K dataset contains numerous users' demographic data. There are 1682 movies in the dataset, with a total of 10,0000 ratings from 943 users. For this evaluation, data were gathered from the https://www.kaggle.com/prajitdatta/movielens-100k-dataset. It consists of the user's age, ID, occupation, and items provided. The datasets are used for 80% of the training, while the remaining 20% is used for testing.

### 4.2. Simulation Setup

The proposed DRWMR system is implemented in python; the initial learning rate is 0.001, and after 1000 iterations, it lowers exponentially by 0.04. The batch size is 200, and the parameter coefficient is 0.01.

### 4.3. Evaluation Criteria

The model's performance is evaluated using six metrics: recall, precision, F1-score, MAE, RMSE, and prediction accuracy.

(i) Recall:
It is the ratio of the total number of relevant recommendations to the actual or true number of relevant recommendations for a new user.
  (19) $$\begin{array}{c} RL=\frac{F_{r}}{T_{r}} \end{array}$$
where *F*_*r*_ denotes the recommendation related to the new user and *T*_*r*_ signifies the real amount of related recommendations.
(ii) Precision:
This metric indicates the precision of the process, i.e., whether the generated recommendations are appropriate for new users.
  (20) $$\begin{array}{c} PN=\frac{F_{r}}{{tot}_{r}} \end{array}$$
where *F*_*r*_ denotes the recommendation related to the new user and *tot*_*r*_ signifies the recommended item's total quantity.
(iii) F1-score:
This score shows the experiment's accuracy based on the recall and precision measures and is calculated by the following equation:
  (21) $$\begin{array}{c} F=\frac{2\times RL\times PN}{PN+RL} \end{array}$$
(iv) RMSE:
It is measured by determining the difference between the predicted and observed values, which is given in the following equation:
  (22) $$\begin{array}{c} R=\sqrt{\frac{1}{Q}}\overset{Q}{\underset{j=1}{\sum }}{\left(k_{j}-{\overset{\wedge }{k}}_{j}\right)}^{2}\text{.} \end{array}$$
(v) MAE:
The magnitude of the difference between the expected and observed values is computed to determine it, which is given in the following equation:
  (23) $$\begin{array}{c} M=\frac{1}{Q}\overset{Q}{\underset{j=1}{\sum }}\left|k_{j}-\hat{K_{j}}\right|\text{,} \end{array}$$
where *Q* signifies the user's total amount, $\hat{K_{j}}$KJ denotes the predicted values, and KJ signifies the observed value.

### 4.4. Comparative Analysis with Existing Methods

The proposed DRWMR system is tested on the movie Lens 100 K dataset, and metrics such as recall, precision, RMSE, MAE, and F1-score are compared to existing approaches such as CTR [17], DDCF [18], CRDTM [19], and HMRNN [22].

#### 4.4.1. Quantitative Analysis

Figure 2 illustrates the RMSE analysis of our proposed DRWMR system with existing methods such as CTR, DDCF, CRDTM, and HMRNN. Our research introduces a novel loss function that minimises the classification loss and ranks pairwise losses. It produces hash codes with high recommendation accuracy and more similar information. Therefore, our proposed DRWMR system reduces the error compared to the existing methods for the top 5, 10, and 15 recommendations. The proposed DRWMR system (0.73) has a low RMSE when compared with existing techniques such as CTR (0.87), DDCF (0.80), CRDTM (0.77), and HMRNN (0.75) for the top 10 recommendations.

Figure 3 shows the MAE analysis. The smallest Hamming distance between the users results in the recommendation to the new user. The weighted Hamming distance is used to determine how similar the users are. So, the errors can be reduced in the recommendation system. The MAE is low for the proposed DRWMR system (0.57) when compared with existing methods such as CTR (0.75), DDCF (0.72), CRDTM (0.705), and HMRNN (0.653) for the top 10 recommendations.

Figures 4 and 5 show the recall and precision analyses. In the proposed DRWMR system, a hash table is built as an additional layer. A table and bitwise weight method are presented based on the performance to attain a better recommendation performance. The proposed DRWMR system assigns weights to various hash bits and hash tables. Also, a hash code is generated based on minimising loss, which can handle users with cold start and sparsity problems. This mechanism attains higher precision and recall. The precision is high for the proposed DRWMR system (0.16) when compared with existing methods such as CTR (0.10), DDCF (0.12), CRDTM (0.129), and HMRNN (0.14) for the top 10 recommendations. The recall is high for the proposed DRWMR system (0.08) when compared with existing methods such as CTR (0.04), DDCF (0.041), CRDTM (0.045), and HMRNN (0.06) for the top 10 recommendations.

Figure 6 shows the *F* − 1 measure analysis. The *F*-measure is high for the proposed DRWMR system (0.101), when compared with existing methods such as CTR (0.06), DDCF (0.064), CRDTM (0.077), and HMRNN (0.08) for the top 10 recommendations.

## 5. Conclusion

The RS has become vital to social networking and business apps such as Flipkart, Amazon, YouTube, and others. Therefore, we introduced the DRWMR system for an accurate recommendation initially. User-item rating data is fed into CNN to extract important features to reduce data sparsity. Then, the hash code is generated by minimising pairwise rank loss and classification loss. A weight is assigned to different hash tables and hash bits. According to weighted Hamming distance, the most similar users were obtained. Finally, the rating of unknown items can be obtained using the weighted average rating of similar users and active users. As a result, we have seen that our proposed DRWMR system performs better in recommending items. The proposed DRWMR system is quantitatively measured by precision (0.16), recall (0.08), RMSE (0.73), MAE (0.57), and F-measure (0.101). It shows better performance in the recommendation system.

## Figures and Tables

**Figure 1:** Architecture of the proposed DRWMR system.

**Figure 2:** RMSE analysis.

**Figure 3:** MAE analysis.

**Figure 4:** Precision analysis.

**Figure 5:** Recall analysis.

**Figure 6:** *F*-measure analysis.

## Data Availability

The datasets generated and analyzed during the current study are available from the corresponding author upon reasonable request.
